The article "Ex-vivo expanded human NK cells express activating receptors that mediate cytotoxicity of allogeneic and autologous cancer cell lines by direct recognition and antibody directed cellular cytotoxicity" was published in 2010. Journal: J Exp Clin Cancer Res.

# Ex-vivo expanded human NK cells express activating receptors that mediate cytotoxicity of allogeneic and autologous cancer cell lines by direct recognition and antibody directed cellular cytotoxicity

**DOI:** 10.1186/1756-9966-29-134

**Published:** 2010-10-11

**Authors:** Caroline J Voskens, Ryuko Watanabe, Sandra Rollins, Dario Campana, Kenichiro Hasumi, Dean L Mann

**Affiliations:** 1 Department of Pathology, University of Maryland School of Medicine, 10 South Pine Street, Baltimore, MD, 21201, USA; 2 Shukokai Clinics, 1-44-6 Asagaya-kita, 166 Tokyo, Japan; 3 Departments of Oncology and Pathology, St. Jude Children's Research Hospital, 262 Danny Thomas Place, Memphis TN 38105, USA

## Abstract

**Background:**

The possibility that autologous NK cells could serve as an effective treatment modality for solid tumors has long been considered. However, implementation is hampered by (i) the small number of NK cells in peripheral blood, (ii) the difficulties associated with large-scale production of GMP compliant cytolytic NK cells, (iii) the need to activate the NK cells in order to induce NK cell mediated killing and (iv) the constraints imposed by autologous inhibitory receptor-ligand interactions. To address these issues, we determined (i) if large numbers of NK cells could be expanded from PBMC and GMP compliant cell fractions derived by elutriation, (ii) their ability to kill allogeneic and autologous tumor targets by direct cytotoxitiy and by antibody-mediated cellular cytotoxicity and (iii) defined NK cell specific receptor-ligand interactions that mediate tumor target cell killing.

**Methods:**

Human NK cells were expanded during 14 days. Expansion efficiency, NK receptor repertoire before and after expansion, expression of NK specific ligands, cytolytic activity against allogeneic and autologous tumor targets, with and without the addition of chimeric EGFR monoclonal antibody, were investigated.

**Results:**

Cell expansion shifted the NK cell receptor repertoire towards activation and resulted in cytotoxicity against various allogeneic tumor cell lines and autologous gastric cancer cells, while sparing normal PBMC. Blocking studies confirmed that autologous cytotoxicity is established through multiple activating receptor-ligand interactions. Importantly, expanded NK cells also mediated ADCC in an autologous and allogeneic setting by antibodies that are currently being used to treat patients with select solid tumors.

**Conclusion:**

These data demonstrate that large numbers of cytolytic NK cells can be generated from PBMC and lymphocyte-enriched fractions obtained by GMP compliant counter current elutriation from PBMC, establishing the preclinical evidence necessary to support clinical trials utilizing autologous expanded NK cells, both directly and in combination with monoclonal antibodies in future cell-based immunotherapy in select solid tumors.

The article "Ex-vivo expanded human NK cells express activating receptors that mediate cytotoxicity of allogeneic and autologous cancer cell lines by direct recognition and antibody directed cellular cytotoxicity" was published in 2010. Journal: J Exp Clin Cancer Res.

## Background

Natural killer cells (NK) were identified more than 30 years ago as a population of lymphokine activated killer cells that showed the ability to kill tumor cells in vitro in the absence of prior immune sensitization of the host [1-4]. Over the ensuing years, much has been learned about regulation of their biologic activity and, in particular, their potential use as an immunotherapeutic modality in cancer [5].

It has become clear that the biologic activity of NK cells is controlled by a complex repertoire of surface receptors which, upon engagement by ligands on a target cell, signal either an inhibitory or activating response [6]. The major inhibitory and activating receptors are products of germ line genes encoding killer cell immunoglobulin-like receptors (KIRs) and in an autologous environment, inhibition of NK cell cytotoxic activity is dominant and governed by epitopes on self HLA class I alleles. In general, cytotoxic activity of NK cells is triggered when the target cell lacks expression of some or all HLA class I molecules; the basis for the "missing self" hypothesis [7].

Recognizing the possibility that NK cells have the ability to kill tumors that lack expression of the inhibitory HLA class I alleles, investigators have reported significant antitumor responses in clinical settings of allogeneic stem cell transplantation. Importantly, clinical effects are demonstrated when inhibitory effects are bypassed by utilizing haplo-identical NK cells and best results are achieved when, in addition, KIR-ligand mismatched NK cells are selected [8,9]. In turn, this approach requires extensive donor screening and careful depletion of allogeneic T cells from the NK cell product before administration to the host in order to avoid the risk of graft-versus-host disease (GvHD) [10].

The possibility that infusion of autologous NK cells could serve as an effective treatment modality for solid tumors has long been considered [11]. However, implementation is hampered by (i) the small number of NK cells in peripheral blood that could be isolated relative to the number of cells that would be required to be effective and the difficulties associated with large-scale production of cytolytic NK cells in compliance with Good Manufacturing Practices (GMP), (ii) the need to activate the NK cells in order to induce NK cell mediated killing of a resident tumor and (iii) the constraints imposed by autologous inhibitory receptor-ligand interactions.

The article "Ex-vivo expanded human NK cells express activating receptors that mediate cytotoxicity of allogeneic and autologous cancer cell lines by direct recognition and antibody directed cellular cytotoxicity" was published in 2010. Journal: J Exp Clin Cancer Res.

The first issue has been addressed in a number of reports that demonstrate that large numbers of NK cells could be expanded from CD56^+ ^cells isolated from peripheral blood mononuclear cells (PBMC) obtained from healthy individuals and patients with hematological malignancies and solid tumors. Expansion was achieved by short term culture with cytokines alone, by cytokines and co-culture with irradiated feeder cells consisting of EBV transformed lymphoblastoid cell lines or cytokines and co-culture with K562 cells that had been transfected with and expresses cell membrane-bound IL-15 and 4-1BBL [12-16]. In most instances, these expanded cells were generated from NK cells (CD56^+^CD3^-^) isolated from peripheral blood using magnetic beads. The expanded NK cells were highly cytotoxic when tested against variety of target cells that consisted primarily of allogeneic cancer cell lines established from hematologic malignancies [12,17].

In addition, a GMP compliant and closed system has successfully been established for the enrichment of monocytes from PBMC using counter current elutriation [18]. Besides a highly enriched population of monocytes, lymphocyte-enriched fractions are also obtained. Currently, clinical studies are ongoing utilizing elutriation derived monocytes for large-scale generation of dendritic cells in order to treat a variety of metastatic cancers.

The objectives of this study were to evaluate if the aforementioned strategies could be combined in order to expand large numbers of NK cells from PBMC from normal individuals and patients with various solid tumors. Furthermore, the possibility to expand NK cells from lymphocyte-enriched cell fractions derived from PBMC by elutriation rather than utilizing isolated CD56^+ ^cells as the starting cell population was determined. In addition, cytolytic allogeneic and autologous activity by direct cytotoxicity as well as antibody-mediated cellular cytotoxicity and NK specific receptor-ligand interactions that mediate target cell killing were defined.

We confirmed that large quantities of cytotoxic NK cells can be expanded from PBMC in the presence of K562 cells expressing membrane-bound IL-15 and 4-1BBLigand from normal individuals and patients with various solid tumors. Ex-vivo expansion tended to alter the balance of NK cell receptor expression towards those that activate and mediate cytotoxicity. This activity resulted in cytotoxicity against various allogeneic tumor targets and more importantly, against autologous-derived gastric tumor targets. Blocking studies identified multiple activating receptor-ligand interactions that would be predicted to mediate NK cell cytotoxicity. Moreover, these activating receptor-ligand interactions were operative in antibody-dependent cellular cytotoxicity (ADCC) in an allogeneic and autologous setting. Importantly, as a mean for future clinical translation, GMP compliant cytolytic NK cells could efficiently be expanded from lymphocyte-enriched cell fractions obtained from PBMC by counter current elutriation.

The article "Ex-vivo expanded human NK cells express activating receptors that mediate cytotoxicity of allogeneic and autologous cancer cell lines by direct recognition and antibody directed cellular cytotoxicity" was published in 2010. Journal: J Exp Clin Cancer Res.

Our studies demonstrate that human NK cells acquire cytolytic activity against autologous gastric tumor cells after ex-vivo expansion and suggest a therapeutic potential for autologous expanded NK cells, both directly and in combination with monoclonal antibodies in future cell-based immunotherapy.

## Methods

### Cells and Cell Fractions

Human blood samples were purchased (BRT Laboratories, Baltimore, MD) and whole peripheral blood mononuclear cells (PBMC) were isolated using density-gradient centrifugation. Using leukapheresis products purchased from the same source, the constitutive cell populations were fractionated by continuous-counterflow elutriation following protocols established by the manufacturer of cell separator (Elutra, Gambro BCT). This instrument uses continuous counter-flow elutriation technology to separate cells fractions based primarily by size and secondarily by specific gravity. In brief, the leukapheresis product was loaded via an inlet pump into a constantly rotating (2400 rpm) elutriation chamber. Based on centrifuge speed and cell density, five elutriated cell fractions were collected. PBMC and various elutriated cell fractions were viably frozen in RPMI-1640 (Invitrogen Corp., Grand Island, NY) supplemented with 20% human AB serum (Gemini Bio-Products, Woodland, CA) and 10% Dimethylsulfoxide (Sigma, St. Louis, MO) using an automated cell freezer (Gordinier Electronics, Roseville, MI) and stored in the vapor phase of liquid nitrogen until used.

The myeloid cell line K562, prostate cancer cell lines LNCaP, PC-3 and DU-145 and breast cancer cell line MCF-7 were available in our laboratory. The lung cancer cell line H358 was kindly provided by Dr. S. Ostrand-Rosenberg (Department of Biological Sciences, University of Maryland Baltimore County, Catonsville, MD) and the Head and Neck cancer cell line TU-167 was kindly provided by Dr. S. Strome (Department of Otorhinolaryngology-Head and Neck Surgery, University of Maryland, Baltimore, MD).

With patient consent and under approval of the Institutional Review Board, peripheral blood mononuclear cells were obtained from 2 patients with gastric cancer undergoing treatment at the Tokyo Clinic and Research Institute. Cell lines (tumor 1 and tumor 2) were established from biopsies of metastatic gastric tumor lesions from the respective patients. All tumor cell lines were cultured in RPMI 1640 supplemented with 10% Fetal Bovine Serum, 1% P/S and 1% Glutamax-1 (cRPMI).

The article "Ex-vivo expanded human NK cells express activating receptors that mediate cytotoxicity of allogeneic and autologous cancer cell lines by direct recognition and antibody directed cellular cytotoxicity" was published in 2010. Journal: J Exp Clin Cancer Res.

### Ex-vivo NK cell expansion

NK cells were expanded from PBMC as previously described with some minor modifications [12]. In brief, PBMC (1.5 × 10^6^) were incubated with irradiated (14,000 rad) K562-mbIL15-41BBL cells (10^6^) in a 24-well tissue culture plate in the presence of 200 IU/ml human IL-2 (R&D Systems Inc) in cRPMI. Half of the culture medium was replaced every 2-3 days with fresh culture medium for the first 6 days. After 6 days of expansion, cells were harvested, washed, counted and re-cultured at a starting cell density of 1 × 10^5^-3 × 10^5^/ml in T-25 or T-75 culture flasks in cRPMI supplemented with IL-2. Cells were expanded for and additional 8 days. Additional cRPMI was added to the flasks if necessary based on cell density.

### Flow Cytometry

Cell surface expression was determined before and after 14 days of cell expansion by staining with directly conjugated mouse anti-human mAb's against CD3, CD56, αβTCR, γδTCR, HLA class I, HLA-DR, Fas, Fas-ligand, KLRD1, NKG2a, KIR3DL1, ILT2, CD62L, KIR3DL2/3, NKG2d, DNAM-1, NKp46, NKp44 and NKp30 (BD Biosciences). Gates were set around NK cells which were defined as CD3^-^CD56^+ ^cells. Surface expression of NK cell ligands was determined on both autologous gastric tumor cell lines and included directly conjugated mouse anti-human nectin-2, PVR, MIC A/B, Fas, HLA class I, HLA class II, HLA-G and purified mouse anti-human HLA-E, ULPB-1, ULBP-2 and ULBP-3. For EGFR-mediated ADCC, gastric tumors were stained with mouse anti-human EGFR mAb. Mouse IgGs were used as isotype controls and purified mAbs were secondarily stained with FITC labelled goat anti-mouse mAb. A minimum of 10000 events were acquired using a BD™ LSR II flow cytometer. Data was analyzed with BD™ FACS DIVA Software.

### Cytotoxicity assays

Cytolytic NK cell activity was measured by 4 hour chromium 51 (^51^Cr)-release assays as previously described [19]. K562 cells were included as target cells in all cytotoxicity assays to assess overall cytotoxicity performance (data not shown). Expanded day 14 cells were purified into separate populations of NK cells (CD3^-^CD56^+^) and NKT/T (CD3^+^CD56^+^/CD3^+^CD56^-^) cells using MACS human CD3 microbeads and non-expanded NK cells were purified from PBMC using a MACS human NK cell isolation kit. (Miltenyi Biotec Inc). Cell purity was determined to be >92% and 95% respectively. To determine ADCC, 10 μg/ml human IgG1 (huIgG1, Sigma-Aldrich Corp, St. Louis, MO, USA) or Cetuximab (University of Maryland Marlene and Stewart Greenebaum Cancer Center Pharmacy) was added to defined wells. Purified mouse IgG1, mouse anti-DNAM-1, NKp46, NKp44, NKp30 or all four together (all at 10 μg/ml) were added to defined wells during 4 hours of cytotoxicity in order to assess specific activating NK cell receptor-tumor ligand interactions. Reduction in cytotoxicity was calculated based on percentage cytotoxicity in the presence of indicate blocking mAb(s) versus percentage cytotoxicity in the presence of mouse control mAb. The % reduction in ADCC was calculated with percentage cytotoxicity in the presence of human IgG1 set at 100%. To minimize changes that may occur when cell lines are established from primary tumors, the gastric cell lines used in these studies were cultured for less than 10 passages after isolation from the primary tumor tissue.

The article "Ex-vivo expanded human NK cells express activating receptors that mediate cytotoxicity of allogeneic and autologous cancer cell lines by direct recognition and antibody directed cellular cytotoxicity" was published in 2010. Journal: J Exp Clin Cancer Res.

### Statistics

Paired two-tailed Student's t tests were used to calculate p values. P < 0.05 was considered to be significant.

## Results

### Cytotoxic NK cells are efficiently expanded from PBMC from normal individuals and patients with various solid tumors without the need of primary enrichment protocols

To achieve large-scale expansion of human NK cells, PBMC were co-cultured in a 1 to 1.5 ratio with lethally irradiated K562 cells expressing membrane-bound IL-15 and 4-1BBLigand (K562-mbIL15-4-1BBL) in culture media containing 200 units IL2/ml. After 14 days of culture, NK cells (CD56^+^CD3^- ^as defined by flow cytometry) expanded greater than 2 orders of magnitude from PBMC (mean 165 fold; range 4-567 fold, n = 6) and cell products became significantly enriched in NK cells (day 0 with mean 7%, range 3.2%-12.6% versus day 14 with mean 45.6%, range 7.4%-76.4%; P = 0.0140). At the same time, NKT cells (CD56^+^CD3^+ ^as defined by flow cytometry) expanded at an average of 57 fold (range 7-234), although no significant enrichment (day 0 with mean 3.8%, range 0.8%-8.1% versus day 14 with mean 11.4%, range 2.3%-17.9%; P = 0.1907) was observed. In contrast, a significant decrease in T cells (CD3^+ ^as defined by flow cytometry) was noted after 14 days of expansion (day 0 with mean 54.5%, range 39.9%-71.2% versus day 14 with mean 30.0%, range 4.2%-58.4%; P = 0.0436) with an absolute expansion of 7 fold (range 2-19). The distribution of NK cells and NKT cells in PBMC after expansion is shown in Figure 1A.

**Figure 1:** **Cytolytic NK cells are efficiently expanded from PBMC**. In the presence of K562-IL15-41BBL **(A) **expanded cells become significantly enriched (P = 0.0307) in NK cells (defined by CD56^+^CD3^- ^cells) after 14 days of culture. Expanded cells were evaluated for cytolytic activity using 4 hour ^51^Cr release assays. Ex-vivo expanded cells from PBMC (■ donor 1 and △ donor 2), but not freshly purified non-expanded NK cells (◇), efficiently lysed allogeneic tumor cell lines derived from breast (MCF-7) and prostate (LNCaP) cancers but not allogeneic or autologous PBMC derived from donor 1 **(B)**. The mean percentage cytotoxicity is shown from triplicate wells. Error bars represent the SD. Lytic activity is likely mediated by NK cells in the expanded cell population (○) since separation in individual populations of NK cells (◇) and NKT/T cells (△) resulted in allogeneic cytolytic activity of the expanded cell population and the purified NK cell population. Little lytic activity was observed in the presence of NKT/T cells alone **(C)**. The mean percentage cytotoxicity is shown from triplicate wells from one representative experiment. Error bars represent the SD. Experiment shown represents one of three individual experiments with three different donors.

The article "Ex-vivo expanded human NK cells express activating receptors that mediate cytotoxicity of allogeneic and autologous cancer cell lines by direct recognition and antibody directed cellular cytotoxicity" was published in 2010. Journal: J Exp Clin Cancer Res.

Importantly, ex-vivo expanded NK cells from healthy donor PBMC efficiently lysed allogeneic breast-and prostate-derived tumor targets but not allogeneic or autologous PBMC (Figure 1B). We did observe that cytotoxicity was associated with overall expansion efficiency. Specifically, the one donor whose cells expanded 4 fold after 14 days of culture demonstrated an average of 11.7% cytotoxicity (effector to target ratio 1:10) against K562 cells whereas donors who expanded an average of 202 fold (range 34-576; n = 4) possessed an average of 59.8% cytotoxicity (range 56.0%-65.9%; n = 4) against K562 cells (data not shown).

Based on CD3 and/or CD56 phenotype, the majority of cells in the expanded cell products represented NK cells while a much smaller proportion represented NKT and T cells (Table 1). To determine if both the NK cells and NKT/T cells mediated cytolytic activity, the two populations were isolated by immunomagnetic bead selection and killing assays against prostate-derived tumor cell targets were performed. Cytolytic activity was mediated by NK cells and not NKT cells (Figure 1C). Interestingly, little to no killing was observed with the NKT/T cell population even though a subpopulation of the T cells was confirmed to be γδ-TCR^+ ^by flow cytometry (data not shown). Although γδ-TCR^+ ^T cells are reported to have lytic activity against allogeneic tumor cells, they first require in vitro activation with isopentenyl pyrophosphate (IPP) and IL-2 [20]. Studies are underway to determine if addition of IPP will expand a cytolytic γδ-TCR^+ ^population.

**Table 1:** Cell phenotype and fold expansion after 14 days of expansion

	**CD3**^**-**^**CD56**^**+ **^**NK cells**		**CD3**^**+**^**CD56**^**+ **^**NKT cells**		**CD3**^**+**^**CD56**^- ^**T cells**	
Donor	Population	Expansion	Population	Expansion	Population	Expansion
	(%)	(fold)	(%)	(fold)	(%)	(fold)
1	7.4	4	17.9	31	58.4	4
2	61.7	140	4.2	26	21.2	9
3	68.5	61	3.1	7	23.1	4
4	76.5	183	2.3	12	4.2	2
5	35.6	576	37.2	234	22.1	19
6	23.9	34	3.8	33	51.2	7
						
Mean:	45.6	165	11.4	57	30.0	7
Range:	7.4-76.5	4-576	2.3-17.9	7-234	4.2-58.4	2-19

The capacity of K562-mb15-41BBL to stimulate expansion of NK cells from peripheral blood of healthy individuals and children with leukemia in remission was previously demonstrated [12,17]. However, there is little information in reference to expand NK cells from PBMC derived from patients with solid tumors. With informed consent, NK cells were expanded from PBMC derived from patients with various solid tumors, including gastric cancer, lung cancer, colon cancer and hepatocellular cancer. After 14 days of culture, cell products became significantly enriched in NK cells (day 0 with mean 23.5%; range 5%-46% versus day 14 with mean 80%; range 60%-95%, n = 6, P = 0.0001 data not shown). Expansion efficiency was comparable between PBMC derived from solid tumor patients versus healthy donor PBMC (mean 316 fold; range 1-1795 with n = 6 versus mean 165 fold; range 4-567 with n = 6, P = 0.6685).

The article "Ex-vivo expanded human NK cells express activating receptors that mediate cytotoxicity of allogeneic and autologous cancer cell lines by direct recognition and antibody directed cellular cytotoxicity" was published in 2010. Journal: J Exp Clin Cancer Res.

These data suggest that NK cells are efficiently expanded from PBMC from normal individuals and more importantly, from patients with various solid tumors without the need of primary enrichment protocols.

### NK cell expansion turns the receptor balance towards activation and results in autologous gastric tumor cell lysis

Human NK cells maintain self tolerance by the expression of at least one inhibitory receptor specific for autologous HLA class I which prevents cytotoxicity against autologous cells [21]. To establish cytotoxicity against autologous target cells, inhibitory signals must be overcome, either by (i) down-regulation of inhibitory ligands on the tumor cell, (ii) enhanced expression of activating receptors on NK cells, (iii) expression of ligands on the tumor target that activate the NK cell or (iv) a combination of thereof. Since NK cell activation is affected by cytokines such as IL-2 and IL-15 [22], we sought to determine if NK cells expanded from PBMC were phenotypically different from non-expanded NK cells (Table 2).

**Table 2:** Phenotypic changes on human NK cells after 14 days of expansion

	Healthy donors (n = 6)					Patient 1		Patient 2	
	Day 0		Day 14						
	Mean (%)	Range (%)	Mean (%)	Range (%)	**P-value**^**a, b **^**(%)**	Day 0	Day 14	Day 0	Day 14
**Activating receptors**									
**DNAM-1**	83	72-90	94	89-97	**0.0335 (↑)**	90	97	37	90
**NKG2D**	83	51-98	96	93-99	0.1074	30	94	87	98
**NKp46**	68	27-91	87	64-97	**0.0161 (↑)**	52	95	19	70
**NKp44**	3	2-5	59	16-93	**0.0039 (↑)**	0,3	29	0,4	15
**NKp30**	52	11-93	82	67-97	**0.0131 (↑)**	7	63	15	70
									
**Inhibitory receptors**									
**KLRD1**	68	56-82	92	86-95	**0.0012 (↑)**	ND	98	49	95
**NKG2A**	46	14-67	68	34-89	**0.00118 (↑)**	ND	84	7	8
**KIR3DL1**	22	10-37	29	17-38	0.1526	ND	21	5	3
**KIR3DL2/3**	28	9-48	29	14-44	0.7858	ND	35	88	96
**LIR1**	22	13-37	6	3-9	**0.0142 (↓)**	ND	18	70	44

^a ^Significant differences (P < 0.05) are indicated in bold

^b ^Arrows indicate significant increase (↑) or significant decrease (↓)

ND; not determined

In expanded NK cells from normal individuals, no significant change was observed in inhibitory receptors KIR3DL1 (P = 0.1526), KIR3DL2/3 (P = 0.7858) and the activating receptor NKG2D (P = 0.1074). In contrast, activating receptors DNAM-1 (P = 0.0061), NKp46 (P = 0.0161), NKp44 (P = 0.0039) and NKp30 (P = 0.0131) were significantly increased in expression after 14 days of expansion. Interestingly, KLRD1 (P = 0.0012) and NKG2A (P = 0.0118), which both form a complex with the inhibitory non-classical HLA class I ligand HLA-E [23,24] were also significantly increased after expansion. Importantly, expression of the inhibitory receptor ILT2 (P = 0.0142) which recognizes multiple HLA class I alleles, including non-classical HLA class I, HLA-G [25], was significantly decreased after expansion.

The article "Ex-vivo expanded human NK cells express activating receptors that mediate cytotoxicity of allogeneic and autologous cancer cell lines by direct recognition and antibody directed cellular cytotoxicity" was published in 2010. Journal: J Exp Clin Cancer Res.

In order to define the ability of expanded NK cells derived from patients with solid tumors to kill their autologous tumors, tumor cell lines were established from tumor biopsies from two metastatic gastric cancer patients undergoing immunotherapy at the Tokyo Clinic and Research Institute. Of note, the expression of inhibitory and activating receptors on expanded NK cells from the gastric cancer donors were generally not different from expression on expanded NK cells from normal donors (Table 2).

Since autologous NK cell cytotoxicity is the net result of engagement of activating NK cell receptors with activating target cell ligands, the two gastric tumor cell lines were first phenotypically characterized for expression of ligands (Table 3) that are known to engage the NK cell receptors identified in table 2. While the ligands for human NKp46, NKp44 and NKp30 are to be defined, both patient cell lines expressed high levels of the inhibitory ligands HLA class I (75% and 67%, respectively) and HLA-G (42% and 57%, respectively) and relatively small amounts of the activation ligands MHC class I chain-related (MIC) A/B (2% and 1%, respectively), UL16 binding protein (ULBP)-1 (both 3%), ULBP-3 (both 3%) and polio-virus receptor (PVR; 8% and 9%, respectively). Importantly, both cell lines expressed the activating ligand nectin-2 (both 92%; specific for DNAM-1) which prompted us to evaluate both cell lines for their sensitivity against autologous NK cells.

The article "Ex-vivo expanded human NK cells express activating receptors that mediate cytotoxicity of allogeneic and autologous cancer cell lines by direct recognition and antibody directed cellular cytotoxicity" was published in 2010. Journal: J Exp Clin Cancer Res.

**Table 3:** Characterization of NK cell ligands on gastric tumor cells

	Patient 1 (N = 2)		Patient 2 (N = 3)	
	Mean	Range	Mean	Range
**Inhibitory ligands**				
**HLA class 1**	75%	71%-80%	67%	30%-97%
**HLA-E**	1%	0%-1%	2%	1%-3%
**HLA-G**	42%	28%-56%	57%	30%-82%
				
**Activating ligands**				
**PVR**	8%	3%-14%	9%	3%-18%
**Nectin-2**	92%	87%-98%	92%	87%-97%
**MIC A/B**	2%	1%-2%	1%	0%-1%
**ULBP-1**	3%	2%-4%	3%	2%-4%
**ULBP-2**	62%	60%-65%	67%	51%-76%
**ULBP-3**	3%	3%-4%	3%	2%-4%
				
**Other**				
**Fas**	36%	21%-50%	95%	88%-99%
**EGFR**	95%	93%-98%	18%	7%-29%

Subsequent 4 hour chromium-release (^51^Cr-release) assays confirmed that gastric tumor cells derived from both patients were killed by autologous expanded NK cells (Figure 2A) and not by resting (non-expanded) NK cells from patient 2. Unfortunately, insufficient numbers of PBMC from patient 1 were available to isolate and test resting NK cells.

**Figure 2:** **Ex-vivo expanded NK cells recognize autologous gastric tumor cells through different activating receptor-ligand interactions**. PBMC from two gastric cancer patients were ex-vivo expanded for 14 days and then tested for cytolytic activity against autologous gastric tumor cells in 4 hour ^51^Cr release assays. **(A) **Ex-vivo expanded cells from both patients (patient 1 and patient 2), but not freshly purified non-expanded NK cells from patient 2, efficiently lysed autologous gastric tumor cells (Effector to Target Ratio 20:1). To evaluate the impact of activating receptor-ligand interactions on autologous tumor cell lysis indicated blocking antibodies (10 μg/ml) were added during 4 hours of incubation. **(B) **Cytotoxicity was reduced in the presence of DNAM-1 (P = 0.0309) and NKp30 (P = 0.0056) for patient 1 and in the presence of NKp46 (P = 0.0003) for patient 2. In both patients autologous cytolytic activity was abrogated in the presence of all four blocking antibodies with P = 0.0111 and P = 0.0001, respectively. Statistical analysis is based on triplicate wells of four (patient 1) and two (patient 2) experiments performed, respectively. Error bars represent the SD. * P < 0.05. MoIgG1 indicates mouse IgG1.

Since expanded NK cells significantly up-regulated DNAM-1, NKp46, NKp44 and NKp30, we performed blocking studies in order to evaluate the importance of these activating receptor-ligand interactions in autologous tumor cell recognition (Figure 2B). As expected, autologous lytic activity was significantly reduced (P = 0.0111 for patient 1 and P = 0.0001 for patient 2) when activating receptor-ligand interactions were interrupted by all four blocking antibodies (mAbs). Specifically, lytic activity of autologous NK cells from patient 1 was significantly reduced in the presence of mAb against DNAM-1 (P = 0.0309) or NKp30 (P = 0.0056) while lytic activity of autologous NK cells from patient 2 was only affected in the presence of mAb against NKp46 (P = 0.003).

The article "Ex-vivo expanded human NK cells express activating receptors that mediate cytotoxicity of allogeneic and autologous cancer cell lines by direct recognition and antibody directed cellular cytotoxicity" was published in 2010. Journal: J Exp Clin Cancer Res.

### Ex-vivo expanded NK cells are capable of autologous and allogeneic target cell lysis by antibody-mediated cellular cytotoxicity

Over many years, it has been postulated that eradication of human tumors may best be accomplished by combining cancer treatments modalities [26,27]. Monoclonal antibodies that react with cell surface structures expressed on cancer cells represent the most successful cancer immunotherapy to date. It is quite clear that their mechanism of action is, at least partially, due to NK cell-mediated ADCC [28]. Since expanded NK cells expressed high levels of CD16 (data not shown), an Fc receptor that mediates ADCC, we sought to determine if lytic activity against the gastric tumor cells could be enhanced in the presence of Cetuximab (Erbitux^®^), a chimeric monoclonal antibody that reacts with the EGFR receptor and is used to treat patients with a variety of solid tumors [29].

Both gastric tumor cell lines were screened for EGFR and only one of the two patient tumor cell lines (patient 1) expressed EGFR (Table 2). Subsequent ^51^Cr-release assays confirmed that allogeneic and autologous cytolytic activity is greatly enhanced in the presence of chimeric anti-EGFR mAb but not in the presence of human IgG1 control antibody (Figure 3A). As expected, the enhancement in cytotoxicity was far more dramatic in the autologous setting if compared to the allogeneic setting since allogeneic tumor cells do not maintain self tolerance through specific inhibitory receptor-ligand interactions.

**Figure 3:** **Cetuximab significantly enhances cytolytic activity and ADCC is negatively affected by inhibition of activating receptor-ligand interactions**. Ex-vivo expanded cells from cancer patient 1 were evaluated for their ability to mediate ADCC against autologous (patient 1) and allogeneic (TU-167 and H-358) EGFR expressing lung cancer cells. **(A) **Cytolytic activity of ex-vivo expanded cells was enhanced in the presence of Cetuximab (10 μg/ml, black bar) but not in the presence of control human IgG1 (10 μg/ml; dotted bar) or media alone (white bar). The mean percentage cytotoxicity is shown from triplicate wells from one representative experiment. Error bars represent the SD. Experiment shown represents one of two individual experiments. **(B) **The addition of blocking antibodies (10 μg/ml) against DNAM-1, NKp46, NKp44 and NKp30 (= all) significantly reduced (P = 0.0176) Cetuximab-mediated ADCC. Statistical analysis is based on three experiments performed. Error bars represent the SD. * P < 0.05. HuIgG1 indicates human IgG1, Ctx; Cetuximab and moIgG1; mouse IgG1.

The article "Ex-vivo expanded human NK cells express activating receptors that mediate cytotoxicity of allogeneic and autologous cancer cell lines by direct recognition and antibody directed cellular cytotoxicity" was published in 2010. Journal: J Exp Clin Cancer Res.

Importantly, the expression of activating receptors on the ex-vivo expanded NK cells positively affected overall cytotoxic activity (Figure 3B) since blocking all four activating receptors on the NK cell surface decreased autologous cytotoxicity if compared with control mAb (P = 0.0176 and P = 0.1019, respectively). These data suggest that the combined strategy of adoptively transferred ex-vivo expanded autologous NK cells with infusion of an mAb that is used for cancer immunotherapy may provide clinical benefit for the treatment of select human solid tumors. To extend these observations, we are attempting to establish cell lines from other solid tumors where PBMC would be available to test NK expansion and direct cytotoxicity and ADCC capability.

### NK cells are efficiently expanded from lymphocyte-enriched cell fractions obtained from PBMC by counter current elutriation

A GMP compliant system has successfully been established for the enrichment of monocytes from PBMC using an Elutra cell separator. In this closed system, PBMC are fractionated by centrifugal elutriation and five cell fractions are obtained. In general, these fractions consist of platelets (fraction 1), erythrocytes mixed with lymphocytes (fraction 2), lymphocytes (fraction 3), lymphocytes mixed with monocytes (fraction 4) and mainly monocytes (fraction 5) as demonstrated in Figure 4 (n = 11). Current clinical cellular therapy protocols use monocytes obtained from elutriated fraction 5 to generate dendritic cells for cancer immunotherapy while the cells from fractions 2, 3 and 4 are usually "archived" in liquid nitrogen. As a means to facilitate clinical translation, we explored the possibility of these GMP compliant cell fractions to serve in future NK cell-based immunotherapy studies. PBMC and separate elutriated cell fractions were expanded with the aforementioned expansion strategy. After 14 days of culture in the presence of K562-mbIL15-41BBL cells and exogenous IL-2, NK cells expanded greater than two orders of magnitude from PBMC (mean 165 fold; range 4-567 fold with n = 6, data not shown), elutriated cell fraction 2 (mean 209 fold; range 3-615 fold with n = 3, data not shown), elutriated cell fraction 3 (mean 131 fold; range 4-339 fold with n = 3, data not shown) and elutriated cell fraction 4 (mean 91 fold; range no expansion-358 fold with n = 4, data not shown). Importantly, expanded cells from PBMC and separate elutriated cell fractions became significantly enriched in NK cells and lysed allogeneic prostate-derived tumor cell lines in a similar fashion (Figure 5A-B). Thus, these data show that large quantities of cytolytic NK cells can be expanded from various elutriated cell fractions collected with the GMP compliant Elutra system.

The article "Ex-vivo expanded human NK cells express activating receptors that mediate cytotoxicity of allogeneic and autologous cancer cell lines by direct recognition and antibody directed cellular cytotoxicity" was published in 2010. Journal: J Exp Clin Cancer Res.

**Figure 4:** **Distribution of lineage-specific phenotypic markers on PBMC and separate cell fractions obtained after counter current elutriation**. PBMC and elutriated cell fractions were stained with various lineage-specific directly-conjugated antibodies and analyzed by flow cytometry **(A)**. Average number of cells and phenotypic distribution (%) expressing lineage-markers in elutriated cell fractions (n = 11) **(B)**.

**Figure 5:** **Ex-vivo expanded cells from elutriated cell fractions efficiently lyse allogeneic prostate cancer cells**. PBMC and elutriated fractions 2, 3 and 4 from the same healthy individual were expanded ex-vivo in the presence of K562-mbIL15-41BBL and IL-2 for 14 days and then tested for *in vitro *cytolytic activity. Cytolytic activity was evaluated in 4 hour ^51^Cr release assays against **(A) **prostate cancer (DU-145, PC-3 and LNCaP) cells. Ex-vivo expanded cells from elutriated cell fractions 2 (◇), 3 (△) and 4 (□) lysed prostate cancer cells in a similar fashion as ex-vivo expanded cells from PBMC (○). **(B) **Elutriated cell fractions become enriched in NK cells (defined by CD56^+^CD3^- ^cells) after 14 days of culture regardless the cellular content of these fractions. The mean percentage cytotoxicity is shown from triplicate wells from one representative experiment. Bars represent the SD. Experiment shown represents one of four individual experiments.

## Discussion

The use of NK cells as a cancer treatment modality in the absence of allogeneic stem cell transplant requires that large quantities of NK cells are generated that kill the tumor cells directly or augment the cytotoxic effect of tumor directed monoclonal antibodies. The critical findings of the studies reported herein are that (i) the technology that was reported to successfully expand NK cells isolated from PBMC [12,17] was also effective in generating large numbers of NK cells from PBMC and various elutriated cell fractions without previous isolation of the CD56^+ ^cells, (ii) activation receptors and other cell surface structures that mediate target cell killing are increasingly expressed on the expanded NK cells, (iii) NK cells expanded from PBMC from patients with solid tumors kill allogeneic and autologous cancer cell lines by direct cytotoxicity and, importantly, mediate ADCC to autologous tumor cell targets in the presence of chimeric mAb and (iv) the interactions of activating receptors DNAM-1, NKp30 and NK-p46 with cognate ligands on the tumor target appear to mediate direct and ADCC mediated autologous cytotoxicity in gastric carcinoma.

The article "Ex-vivo expanded human NK cells express activating receptors that mediate cytotoxicity of allogeneic and autologous cancer cell lines by direct recognition and antibody directed cellular cytotoxicity" was published in 2010. Journal: J Exp Clin Cancer Res.

For translation into the clinic it is important to observe that besides NK cells, relatively small numbers of NKT and T cells are expanded in this system. These cell populations may mediate GvHD when infused together with NK cells in adoptive allogeneic immunotherapy protocols. GvHD is a serious, potentially life-threatening, condition resulting from transplanted or infused allogeneic donor cell recognition of the recipients' tissues as non-self, and is predominantly mediated by CD3^+ ^T cells [30]. These cells are often depleted to prevent GvHD, as could be accomplished with the cells expanded by the protocol presented here. Depletion of T cells from the NK cell product before administration to the host is likely to be less critical in the autologous setting.

An important observation in our studies was that the expanded NK cells did not kill autologous and allogeneic PBMC, an indication that despite the increase in surface expression of activating receptors on the NK cells, the inhibitory ligands expressed on normal PBMC were dominant and able to control cytolytic activity against non-malignant cells. This is further illustrated in that both gastric tumor cell lines were susceptible to autologous cytotoxicity despite the expression of high levels of inhibitory classical and non-classical HLA class I molecules. These data suggest that, under certain conditions, activating receptor-ligand recognition may override receptor-ligand interactions that inhibit NK activity. Emerging data indicates that important triggers in this interaction are surface structures (ligand) that are expressed on cells that have undergone malignant transformation. In addition, it is well recognized that HLA class I expression the major NK cell inhibitory structure, is often down regulated in many solid tumors. In the case of autologous NK cell cytotoxicity against PBMC, inhibitory signals still predominated over activating signals, since no cytotoxicity of NK cells against autologous or allogeneic PBMC was observed. Our results indicate that the NK cells expanded and activated by the methods described do not recognize and kill non-transformed cells.

In addition, while significantly higher levels of the inhibitory CD94/NKG2A complex were expressed after ex-vivo cell expansion, it did not affect the potential of autologous gastric tumor cell recognition. The CD94/NKG2A complex is reported to directly inhibit NK cell cytotoxicity through recognition of HLA-E [31]. Although both autologous gastric tumor cell lines did not express HLA-E (Table 3), we can not rule out that autologous tumor cell recognition will not be affected in HLA-E expressing tumors.

The article "Ex-vivo expanded human NK cells express activating receptors that mediate cytotoxicity of allogeneic and autologous cancer cell lines by direct recognition and antibody directed cellular cytotoxicity" was published in 2010. Journal: J Exp Clin Cancer Res.

The ligands for natural cytotoxicity receptors NKp30, NKp44 and NKp46 are currently unknown. However; we postulate that at least NKp46 and NKp30 may be involved in autologous gastric tumor cell recognition since lytic activity was abrogated in the presence of blocking antibody against these receptors. Since no significant change was observed in NKG2D expression on expanded NK cells, we did not directly test the involvement of this activating receptor in autologous gastric tumor cell cytotoxicity. The fact that autologous cytotoxicity was not completely inhibited by a combination of anti-DNAM-1, NKp46, NKp44 and NKp30 may indicate that NKG2D or other unidentified receptors may also be involved. Importantly, the interaction between NK cell receptors and their ligands has recently been shown to abrogate NK cell mediated cytotoxicity of human and mouse melanoma cell lines [32].

Of note, both tumor cell lines also expressed high levels of Fas which is recognized to establish cell death upon interaction with its ligand, Fas-ligand [33]. In order to test the possibility of target cell-induced killing of the expanded NK cells, all NK cells were evaluated for Fas and Fas-ligand expression before and after ex-vivo expansion. Although expanded NK cells up-regulated high levels of Fas, they did not express Fas-ligand (data not shown).

It has been suggested that in order to overcome self tolerance, multiple activating receptor-ligand interactions should be engaged [31]. Indeed, multiple activating interactions appear to be involved in autologous cytotoxicity of tumor cells derived from patient 1 when the inhibition of cytotoxicity, in the presence of all 4 antibodies, is compared with DNAM-1 or NKp30 alone (P = 0.0356 and P = 0.0165, respectively). In contrast, no significant additional decline in autologous cytotoxicity was observed for patient 2 when cytolytic activity of all four activating receptors was compared to NKp46 alone (P = 0.7359). We postulate that these data reflect variation in expression of receptor-ligand combination in humans that are known to be operative in the control of NK cell cytotoxic activity. These variations include HLA and KIR polymorphism as well as tumor type and tumor origin (e.g. primary versus metastatic tumor cells). This is illustrated in a recent report on studies in patients with multiple myeloma [34] where the investigators demonstrated no specific association of autologous NK cell cytotoxicity with a single activating NK cell receptor. In fact, autologous cytotoxic effects were more likely mediated by several activating NK cell receptors which is also in agreement with a previous report [35] demonstrating that natural cytotoxicity of resting NK cells requires co-activation by more than one receptor.

The article "Ex-vivo expanded human NK cells express activating receptors that mediate cytotoxicity of allogeneic and autologous cancer cell lines by direct recognition and antibody directed cellular cytotoxicity" was published in 2010. Journal: J Exp Clin Cancer Res.

While currently elutriated cell fraction 5 is used for monocyte and dendritic cell-based immunotherapy therapy protocols [36,37], we demonstrated that cytolytic NK cells can be expanded from elutriated cell fractions 2, 3 and 4 regardless of the cellular content of these fractions. However, since NK cell expansion from fraction 4 failed in two out of four experiments, while expansion from PBMC and elutriated cell fractions 2 and 3 was highly successful, and considering the relative high amount of erythrocytes in fraction 2, it may be best to primarily utilize fraction 3 in NK cell expansion protocols. Of note, variability in expansion rates between donors is observed and requires further testing to determine the extent of this variation in the general population. Overall, these data provide a foundation for the large-scale generation of cytolytic NK cells from elutriated cell fractions, which could be employed alone or in combination with other cellular components such as dendritic cells for application in cellular therapy of cancer.

## Conclusions

In summary, the large amount of cytotoxic NK cells generated by this ex-vivo expansion protocol provides the numbers of NK cells that will probably be required to be effective in the case of a large tumor burden. The ability of the expanded cells to mediate ADCC offers the possibility that their effect may be amplified if given in conjunction with a cancer cell directed mAb. An important issue to address is the ability of adoptively transferred NK cells to home and infiltrate into solid tumor tissue. Although the expanded NK cells only expressed small amounts of CD62L (data not shown), which is associated with homing into secondary tissue, we postulate that trafficking into the tumor micro-environment may be enhanced by opsonizing tumor cells with chimeric antibody. Clinical studies are needed to confirm this hypothesis, as well as to establish the therapeutic benefit of infusion of large number of ex-vivo expanded autologous NK cells.

## Competing interests

The authors declare that they have no competing interests.

## Authors' contributions

CJV participated in the design of the experiments, conducted laboratory studies, prepared figures and tables and drafted the manuscript. RW established gastric tumor cell lines. SR conducted laboratory studies and assisted in the manuscript preparation. DC provided the transfected cell line and advice on NK cell expansion. KH cared for patients in the study and biopsied tissue. DLM oversaw the entirety of the project and assisted in the manuscript preparation. All authors read and approved the manuscript.
